# *In Silico* Characterization of an Important Metacyclogenesis Marker in *Leishmania donovani*, HASPB1, as a Potential Vaccine Candidate

**DOI:** 10.1155/2023/3763634

**Published:** 2023-06-07

**Authors:** Bahareh Kordi, Esmaeil Roohparvar Basmenj, Hamidreza Majidiani, Gholam Basati, Dariush Sargazi, Naser Nazari, Morteza Shams

**Affiliations:** ^1^Department of Agricultural Science, Technical and Vocational University (TVU), Tehran, Iran; ^2^Biophysics Department, Faculty of Biological Sciences, Tarbiat Modares University, Tehran, Iran; ^3^Department of Basic Medical Sciences, Neyshabur University of Medical Sciences, Neyshabur, Iran; ^4^Healthy Aging Research Centre, Neyshabur University of Medical Sciences, Neyshabur, Iran; ^5^Zoonotic Diseases Research Center, Ilam University of Medical Sciences, Ilam, Iran; ^6^Veterinary Medicine, Zabol Veterinary Network, Zabol, Sistan and Baluchistan, Iran; ^7^Department of Parasitology and Mycology, School of Medicine, Kermanshah University of Medical Sciences, Kermanshah, Iran

## Abstract

Visceral leishmaniasis is a life-threatening infectious disease worldwide. Extensive experiments have been done to introduce potential vaccine candidates to combat leishmaniasis. The present study was done to evaluate *Leishmania donovani* hydrophilic acylated surface protein B1 as a potential vaccine candidate using *in silico* methods. For this aim, server-based predictions were performed regarding physicochemical characteristics, solubility, antigenicity, allergenicity, signal peptide, transmembrane domain, and posttranslational modifications (PTMs). Also, secondary and tertiary structures were predicted using NetSurfP-3.0 and I-TASSER, respectively. The 3D model was further subjected to refinement and validation, and promising B-cell, cytotoxic T-lymphocyte (CTL; human, dog), and helper T-lymphocyte (HTL; human) epitopes were predicted. The protein had a molecular weight of 42.19 kDa, with high solubility (0.749), stability (instability index: 21.34), and hydrophilicity (GRAVY: -2.322). No signal peptide or transmembrane domain was predicted, and the most abundant PTMs were phosphorylation, O-glycosylation, and acetylation. Many coils and disordered regions existed in the secondary structure analysis, and the tertiary model had a good confidence score (-0.79). Next, the ProSA-web and PROCHECK tools showed adequate improvements in the refined model compared to the crude model. Only 4 shared B-cell epitopes among three web servers (ABCpred, BepiPred 2.0, and SVMTriP) were shown to be antigenic, nonallergenic, and with good water solubility. Also, five potent CTL epitopes in dogs and five in humans were predicted. Notably, two HTL epitopes were found to be potential IFN-*γ* inducers. In conclusion, our results demonstrated several immunogenic epitopes in this protein, which could be directed towards multiepitope vaccine design.

## 1. Introduction

Leishmaniases are a group of vector-borne diseases that threaten about 350 million people in 98 countries and have been classified as one of the six major neglected tropical diseases (NTDs) worldwide [1]. The protozoan parasites of the genus *Leishmania* (family Trypanosomatidae) are known as the causative agents, being transmitted through biting by female phlebotomine sandflies, i.e., *Phlebotomus* and *Lutzomyia*, in the Old World and New World, respectively [2]. The *Leishmania* parasites are obligatory intracellular organisms with two common interchangeable forms: nonflagellated amastigotes within particular immune cells (macrophages and dendritic cells) and flagellated promastigotes within the sandfly gut. This parasitic infection manifests in three important clinical forms, including cutaneous leishmaniasis (CL), mucocutaneous leishmaniasis (MCL), and visceral leishmaniasis (VL) [3]. In many areas, CL is recognized as the most widespread type of the infection, with a particular impact on 0.7-1.2 million individuals, mostly in the Americas, Central Asia, the Middle East, and the Mediterranean Basin [4], whereas VL (so-called as kala-azar) is the most severe form with an incidence rate of 50,000 to 90,000 individuals annually, particularly in Brazil, eastern Africa, and the Indian subcontinent. *Leishmania donovani* (*L. donovani*) and *L. infantum* are known as the principal agents of VL [4, 5].

The VL control strategies have remained unsatisfactory in different endemic areas, possibly due to inadequate vector (sandflies) and/or reservoir (mostly canids) control, along with limited treatment options [6]. First-line therapies such as pentavalent antimonials and amphotericin B are costly and may incur severe toxic effects, including cardiotoxicity, nephrotoxicity, and hepatotoxicity. These compounds are needed to be administered at long-term intervals and may, also, be well tolerated by drug-resistant parasites, causing treatment failure [7, 8]. On this premise, vaccine development seems to be a safer option to effectively control VL infections in endemic areas.

With the advances in genome sequencing technologies and computer sciences, various biomedical databases and computational methods were developed, which increased our knowledge of host-pathogen interactions at the molecular level; this can be advantageous to vaccinology related studies against infectious zoonotic diseases such as VL [9]. In other words, such information enables us to detect, organize, and generate novel antigenic proteins and promiscuous B- and T-cell epitopes in order to devise rational next-generation vaccine candidates in a cost- and time-effective manner [10]. In this sense, several multicomponent vaccine candidates such as the putative Q protein, Leish110-f, Leish111-f, and KSAC have shown protective immune responses [11–13]. A potent vaccine candidate against *Leishmania* would be capable of strong stimulation of IFN-*γ*-producing helper type-I T-cells (Th1) via antigen-presenting cells (APCs), resulting in macrophage activation and a subsequent upsurge in nitric oxide (NO) and reactive oxygen species (ROS) to encounter infective amastigotes [14]. Previously, several *Leishmania* antigens have been introduced and used in vaccination studies [15]. The hydrophilic acylated surface proteins (HASPs) are encoded by chromosome 23, originally called the LmcDNA16 locus [16], in all *Leishmania* species [17]. Among these, HASPB has been in focus and is expressed on the plasma membrane of metacyclic promastigotes as well as amastigotes [18]. It has been shown to be highly immunogenic, demonstrating durable immunity in canine models of *L. donovani* infections [19]. The present study was done to characterize some of the physicochemical and structural properties along with immunogenic epitopes of the *L. donovani* HASPB1 (LdHASPB1) using several immunoinformatic approaches.

## 2. Methods

### 2.1. Amino Acid Sequence Retrieval

The amino acid sequence of the LdHASPB1 protein was retrieved in an FASTA format through a leading high-quality, comprehensive, and freely accessible resource of protein sequences and functional information, UniProt Knowledge Base [20], available at https://www.uniprot.org/,under accession number O77301_LEIDO.

### 2.2. Forecasting Basic Antigenic, Allergenic, Solubility, and Physicochemical Characteristics of LdHASPB1

Some of the preliminary physicochemical properties of the protein were predicted using the ExPASy ProtParam web tool (https://web.expasy.org/protparam/) [21]. The server performs a prediction to evaluate the instability index, aliphatic index, grand average of hydropathicity (GRAVY), estimated half-life, amino acid composition, theoretical isoelectric point (pI), and molecular weight (MW). The protein solubility was evaluated using the Protein-Sol web tool, developed by the University of Manchester (https://protein-sol.manchester.ac.uk/). “The server provides a fast, easy-to-use, sequence-based method for predicting protein solubility based on the population average for the experimental *Escherichia coli* (*E. coli*) dataset,” and values above 0.45 are good soluble proteins [22]. The antigenicity of the LdHASPB1 protein was demonstrated by using the VaxiJen v2.0 web server, available at http://www.ddg-pharmfac.net/vaxijen/VaxiJen/VaxiJen.html, which performs an alignment-independent prediction of protective antigens with 70-89% accuracy [23]. Regarding antigenicity prediction by the VaxiJen v2.0 server, “parasite” was selected as the target organism, and the threshold of prediction was set at 0.45. Finally, the allergenicity of the protein was determined using a hybrid approach of the AlgPred v2.0 online server (https://webs.iiitd.edu.in/raghava/algpred2/), employing random forest (RF), basic local alignment search tool (BLAST), and Multifocal Electroretinogram Classification Interface (MERCI) machine learning techniques [24].

### 2.3. Signal Peptide, Transmembrane Domain, Subcellular Localization, and Posttranslational Modification (PTM) Site Prediction

A number of PTM sites were predicted for the LdHASPB1 protein, including palmitoylation [25], phosphorylation [26], O-glycosylation [27], and N-glycosylation [27] as well as lysine acetylation [28]. For this aim, multiple online tools from DTU Health Tech Services (NetPhos 3.1, NetOGlyc 4.0, and NetNGlyc 1.0) (https://services.healthtech.dtu.dk) and the Cuckoo workgroup (CSS-Palm and GPS-Pail 2.0) (http://biocuckoo.org/) were used. Furthermore, regarding the prediction of signal peptide, transmembrane domain, and subcellular localization of eukaryotic proteins, the SingalP-6.0 [29], Deep TMHMM [30], and DeepLoc2.0 [31] online tools, available at https://services.healthtech.dtu.dk, were utilized, respectively.

### 2.4. Secondary and Tertiary Structure Predictions

The structural analysis of the protein was initially done using secondary structure prediction by the NetSurfP-3.0 server (https://services.healthtech.dtu.dk/service.php?NetSurfP-3.0). This server predicts the surface accessibility, secondary structure, disordered regions, and phi/psi dihedral angles of residues in a particular amino acid sequence [32]. Subsequently, a fully automated protein homology modelling tool, Iterative Threading ASSEmbly Refinement (I-TASSER), was used to predict the top-five three-dimensional (3D) models of the protein using derived structural templates using the multiple threading approaches of the local metathreading server, LOMETS [33]. The I-TASSER server is accessible at https://zhanggroup.org/I-TASSER/. The validity of each model relies on a confidence score (*C*-score) ranging between -5 and 2, where a higher *C*-score usually represents a more confidently predicted model [33].

### 2.5. Refinement and Validation of the 3D Model

The best-predicted 3D model (highest *C*-score) was further subjected to the GalaxyRefine web server for relaxation and energy minimization in the final model. The CASP10 refinement method is employed by this server for side chain reestablishment and repacking by molecular dynamic simulation at the whole protein structure level [34]. Next, the refined 3D model of the LdHASPB1 protein was submitted to a number of web tools for validation, including ProSA-web and PROCHECK. Based on the ProSA-web server, a *Z*-score is assigned to each input structure that is comparable to that of naïve proteins with the same conformation and size; the *Z*-score is defined as “energy separation between the native fold and the average of an ensemble of misfolds” [35]. The PROCHECK web tool evaluates the stereochemical quality of a protein structure through a residue-by-residue geometry analysis and illustrates the phi-psi torsion angles for each amino acid in allowed and disallowed regions, known as the Ramachandran plots [36].

### 2.6. Prediction of Continuous and Conformational B-Cell Epitopes

Continuous B-cell epitopes were predicted using a multimethod approach, so three web servers were initially employed, including ABCpred (http://webs.iiitd.edu.in/raghava/abcpred), BepiPred-2.0 (https://services.healthtech.dtu.dk/service.php?BepiPred-2.0), and SVMTriP (http://sysbio.unl.edu/SVMTriP/) servers. The ABCpred server performs prediction based on a recurrent neural network (RNN) [37], while support vector machine- (SVM-) based prediction through tri-peptide similarity and propensity score combination (SVMTriP) is done by the SVMTriP server [38]. Also, “BepiPred-2.0 is based on a random forest (RF) algorithm trained on epitopes annotated from antibody antigen protein structures” [39]. Subsequently, those linear B-cell epitopes shared among the outputs of the servers were further screened in terms of antigenicity, allergenicity, and water solubility via the VaxiJen v2.0, AllerTOP v2.0 (http://www.ddg-pharmfac.net/AllerTOP), and PepCalc (http://www.pepcalc.com) web servers, respectively. In addition, conformational B-cell epitope prediction was accomplished using the ElliPro tool of the IEDB web server, with a substantial area under the curve (AUC) score of 0.732 and default settings of 6 Å max distance and 0.5 min score [40].

### 2.7. Prediction and Screening of Helper T-Lymphocyte (HTL) and Cytotoxic T-Lymphocyte (CTL) Epitopes

Those epitopes with specific affinity to the class II major histocompatibility complex molecules (MHC-II), which are known as HTL epitopes, were predicted using the MHC-II epitope prediction tool of the IEDB web server by the selection of the recommended prediction method, “Human” as the target host, and the “HLA reference set alleles” option (population coverage over 97%) [41]. The top 10 epitopes with lower percentile ranks (higher binding affinity) were further screened regarding antigenicity, allergenicity, and interferon-gamma (IFN-*γ*) induction by using the VaxiJen v2.0, AllerTOP v2.0, and IFNepitope (http://crdd.osdd.net/raghava/ifnepitope/) online tools, respectively. The latter employs a dataset of MHC-II-binding IFN-*γ*-inducers and noninducers, and the most accuracy can be reached by selecting a hybrid model (>81.39%) [42], as we did here. The hybrid approach is a combination of motif-based and machine learning-based approaches; based on Dhanda et al. [42] [42], “First of all, the sequences were separated that could be correctly predicted via motif-based approach and the remaining sequences were then predicted using SVM. Finally, the performance was evaluated by adding the truly predicted peptides from the motif-based method with SVM-based predictions.”

Those 9-10-mer CTL epitopes (MHC-I binders) specific to humans were predicted using the IEDB MHC-I epitope prediction tool, available, using the IEDB recommended method 2020.09 (NetMHCpan EL 4.1) [41]. This prediction was done with the selection of a reference HLA allele set, including 16 class A alleles (01 : 01, 02 : 01, 02 : 03, 02 : 06, 03 : 01, 11 : 01, 23 : 01, 24 : 02, 26 : 01, 30 : 01, 30 : 02, 31 : 01, 32 : 01, 33 : 01, 68 : 01, and 68 : 02) and 11 class B alleles (07 : 02, 08 : 01, 15 : 01, 35 : 01, 40 : 01, 44 : 02, 44 : 03, 51 : 01, 53 : 01, 57 : 01, and 58 : 01) [43]. Those epitopes with a higher binding affinity (percentile rank < 1) [41] were screened in terms of antigenicity (VaxiJen v2.0) and allergenicity (AllerTOP v2.0). Moreover, high-affinity epitopes for dog leukocyte antigen (DLA) class-I molecules (i.e., DLA-8803401, DLA-8850101, and DLA-8850801) were predicted using the abovementioned tool in IEDB, with subsequent antigenicity (VaxiJen v2.0) and allergenicity (AllerTOP v2.0) screening.

## 3. Results

### 3.1. Antigenicity, Allergenicity, Solubility, and Physicochemical Profiles of LdHASPB1

The VaxiJen antigenicity score for the LdHASPB1 protein was calculated to be 1.4409, rendering it a highly antigenic molecule. Based on the AlgPred server output, this protein possesses no allergenic traits, whereas it was shown to be highly soluble, according to the 0.749 solubility score predicted by the Protein-Sol online tool. The ExPASy ProtParam tool provided a number of important physicochemical characteristics for the examined protein; the output of this server demonstrated that the protein possesses 401 amino acid residues in length, with an MW of 42.19 kDa and a pI of 4.64. Moreover, there were about two-fold more negatively charged residues (Asp + Glu) in the sequence (*n* = 106) than positively charged ones (*n* = 53). The half-life of LdHASPB1 in mammalian reticulocytes was over 30 hours, and the protein was demonstrated to be low thermotolerant (aliphatic index: 5.89), stable (instability index: 21.34), and an extremely hydrophilic molecule (GRAVY: -2.322) (Table 1).

### 3.2. Forecasting Signal Peptide, Transmembrane Domain, Subcellular Localization, and PTM Sites

No signal peptide or transmembrane domain was detected in the LdHASPB1 protein sequence, based on the SignalP and DeepTMHMM web servers, respectively. Additionally, the DeepLoc tool revealed that the protein is probably a cell membrane component (likelihood: 0.63). N-Glycosylation and palmitoylation sites were rarely predicted in the protein sequence, whereas lysine acetylation, O-glycosylation, and phosphorylation sites were abundantly predicted in the LdHASPB1, with 11, 16, and 28 regions, respectively. The detailed properties of the PTM sites are provided in Table 1.

### 3.3. Secondary Structure Analysis

The residues were exposed in most parts of the sequence, according to the NeteSurfP-3.0 server, with frequent coil regions. Also, there observed a high probability of disordered regions throughout the protein sequence (Table 1 and Figure 1).

### 3.4. Tertiary Structure Prediction, Refinement, and Validation

A powerful homology modelling web server, I-TASSER, was employed for the 3D illustration of the LdHASPB1 protein. This structure-based prediction is performed by using similar templates, and the server finally provides the best five models. In the present study, models with *C*-scores of -0.79 (model 1), -2.84 (model 2), -2.99 (model 3), -3.88 (model 4), and -4.16 (model 5) were predicted. Pertinent to a higher *C*-score in model number 1 (estimated TM-score: 0.61 ± 0.14, estimated root-mean-square deviation (RMSD): 8.6 ± 4.5 Å) (Table 1 and Figure 2), it was selected as the best model and further refined it using the GalaxyRefine web server. The output of GalaxyRefine was five refined models with different global distance tests (GDT-HA), RMSD, MolProbity, clash score, poor rotamers, and Rama favored; based on the highest GDT-HA, RMSD, MolProbity, lower clash score, poor rotamers, and Rama favored, model number four was selected here with qualification scores of 0.9202, 0.504, 2.335, 10.7, 1.3, and 82.2, respectively. The ProSA-web results confirmed the improvements in the final refined 3D model (*Z*-score: -1), in comparison with the crude model (*Z*-score: -0.77) (Figure 3). Based on the Ramachandran plot analysis, 165 (56.3%) of residues in the crude model were appointed to the most favored regions, followed by 91 (31.1%), 22 (7.5%), and 15 (5.1%) of residues in the additional allowed, generously allowed, and disallowed regions, respectively. After refinement, 216 (73.7%), 55 (18.8%), 8 (2.7%), and 14 (4.8%) of the residues were allocated to the most favored, additional allowed, generously allowed, and disallowed regions, respectively (Figure 4).

### 3.5. Linear and Conformational B-Cell Epitopes of LdHASPB1

In this study, three different methods of prediction were used for linear B-cell epitopes using the ABCpred, BepiPred-2.0, and SVMTriP web tools, with strict thresholds. The output of each server was compared with that of two others; shared epitopes were extracted and screened. On this basis, among the 8 common linear B-cell epitopes, 4 were shown to possess good antigenicity, no allergenicity, and with good water solubility, based on the VaxiJen, AllerTOP, and PepCalc servers, respectively. These epitopes were as follows: “TQKNDGDG,” “KEDGHTQK,” “AQEKNEDGHNVGD,” and “GDGPKEGENLQ” (Table 2). Also, three conformational B-cell epitopes were predicted for the LdHASPB1 protein using the ElliPro tool, as follows: (i) 14 residues, score: 0.802; (ii) 107 residues, score: 0.695; and (iii) 105 residues, score: 0.679. More details are illustrated in Figure 5.

### 3.6. Prediction and Screening of Potent HTL and CTL Epitopes

Human HTL epitopes were predicted using the IEDB MHC-II tool and the HLA reference set. The server output included top-ten epitopes with lower percentile ranks, which were further screened in terms of antigenicity, allergenicity, and IFN-*γ* induction. Only two epitopes, including “EANHGGATGVPPKHT” and “TEANHGGATGVPPKHT,” possessed good antigenicity and positive IFN-*γ* induction without allergenicity (Table 3). Also, several human MHC-I binders were predicted using the reference HLA alleles and a strict threshold for percentile rank (<1), which were further screened for antigenicity and allergenicity. Among these, five epitopes were shown to possess antigenicity and were nonallergenicity, encompassing “EANHGGATGV,” “EPQKRADNI,” “SAKEPQKRA,” “APKEDGHTQ,” and “EPQKRADNI” (Table 4). In addition, regarding the DLA class-I binding, five epitopic regions were predicted with high antigenicity and nonallergenic, including “KDSAKEPQKR” (DLA-8803401), “EANHGGATGV,” and “KTTEANHGGA” (DLA-8850101) as well as “KDSAKEPQKR” and “TQKNDGDGPK” (DLA-8850801) (Table 5).

## 4. Discussion

Vaccination appears to be the best mainstay in controlling *Leishmania*-induced infections such as kala-azar [44]. An efficacious vaccine candidate against leishmaniasis is anticipated to elicit functional and protective immune responses by igniting the leishmanicidal properties of macrophages, hence preventing the increase in parasite load and subsequent pathological immune imbalance [45]. So far, different vaccination strategies have been used to design vaccines that prevent human and/or canine leishmaniasis [5]. Subunit vaccines are of particular interest among others since they carry immunogenic components of a given pathogenic organism. Thus, they are safer than killed/attenuated vaccines and induce more specific and targeted immune stimulation [46]. In this sense, immunoinformatic-based web servers and online tools can assist us in discovering novel vaccine targets in a considerable amount of genomic and proteomic data, facilitating rational vaccine design [47]. As mentioned before, *Leishmania* HASPs possess a stage-regulated expression pattern, only being confined to metacyclic promastigotes and amastigotes [18]. They are highly immunogenic proteins so that sera of VL- and CL-infected can efficiently detect recombinant HASPB (rHASPB) protein [48, 49]. HASPB is, also, a metacyclogenesis marker in the sandfly vector [17]. The ubiquity of HASPs in all tested *Leishmania* species is beneficial for producing a general leishmaniasis vaccine [50, 51]; hence, it deserves further exploration through a set of *in silico* methods. In the current study, *in silico* characterization and prediction of B- and T-cell epitopes of the LdHASPB1 protein, as a potential vaccine candidate, were performed using immunoinformatic web servers.

In the first step, the biochemical characteristics of LdHASPB1 were evaluated using a set of bioinformatics web servers. This 401-residue protein had an MW of about 42 kDa, and most of its residues were negatively charged (Asp + Glu). Reportedly, charged residues in a protein sequence play a significant role in protein orientation/position [52], and abundant negatively charged ones preferentially occur at the noncytoplasmic flank [53]. In this study, the pI of the LdHASPB1 protein was estimated to be 4.64. A pI is a charge at which the pH turns zero so that in pH ranges above and below the pI, a given protein would be negatively charged and positively charged, respectively [54]. The protein instability index (21.34) showed that the protein is stable in an experimental test tube. Moreover, a GRAVY score of -2.322 and an aliphatic index of 5.89 showed that the LdHASPB1 protein is a fully hydrophilic and weak thermotolerant molecule, respectively. The relative volume of a protein occupied by its aliphatic side chains (alanine, valine, leucine, and isoleucine) is termed as an aliphatic index, enabling the protein to be thermostable in a wide range of temperatures [55]. Although a low aliphatic index was predicted for this protein, the main focus of this study was on the extensive epitope mapping of LdHASPB1, which can be used towards multiepitope vaccine construction against VL cases in humans and dogs. The GRAVY score is an estimated mean of hydrophilicity and hydrophobicity values for individual residues, so scores over or below zero indicate hydrophobicity and hydrophilicity, respectively [56]. In addition, this protein was shown to be highly antigenic and nonallergenic with high solubility. Understanding such preexperimental chemical and biophysical properties is necessary for future wet-lab experiments. Of the predicted PTM sites, phosphorylation was the most frequent with 28 regions, followed by O-glycosylation sites (16) and lysine acetylation regions (11). It is said that these PTM sites are decisive in recombinant protein production, so eukaryotic expression systems (yeast, insect, or mammalian) are more preferred than bacterial hosts to produce those proteins having different PTM sites [57]. Since the protein was predicted to be destined for the cell membrane using the DeepLoc server, neither a signal peptide nor a transmembrane domain existed, according to the SignalP-6.0 and DeepTMHMM servers, respectively.

Using the NetSurfP-2.0 server, surface accessibility, secondary structure, and disordered regions were predicted in the submitted protein sequence. The output showed that almost all regions of the protein were structurally disordered and surface accessible in nature. Disordered proteins are highly abundant and mostly dedicated to regulatory functions and molecular signaling. Supposedly, these regions are likely immunological targets for antibodies; hence, they seem to be important in vaccination studies [58]. Also, exposed surfaces in a protein facilitate the process of epitope mapping by specific antibodies [59]. Random coils were the only secondary structure predicted and have been considered as randomly oriented polymer conformation bonded to nearby units [60]. In general, the protein conformation is maintained and protected during molecular interactions using internally located structures such as coils. Based on the I-TASSER server, pair-wise structure similarity reported five models, among which the first model with the highest *C*-score (-0.79) was selected with a TM-score of 0.61 ± 0.14 and an estimated RMSD of 8.6 ± 4.5 Å. The 3D model was further subjected to refinement and validation. According to the ProSA-Web and PROCHECK analyses, the quality of the refined model was enhanced after refinement as compared with the crude model.

Acquired immune responses play a major role in the prevention and/or control of *Leishmania*-induced infection in susceptible hosts. During the metacyclic phase, the HASPB1 protein can be exposed to the plasma membrane surface, facilitating detection by specific antibodies [18]. On this basis, we predicted linear and conformational B-cell epitopes for the LdHASPB1 protein. A multistep approach was conducted to screen shared linear B-cell epitopes using six web servers; three were used for the identification of shared linear B-cell epitopes (BepiPred-2.0, ABCpred, and SVMTriP), and three were exploited for screening in terms of antigenicity, allergenicity, and water solubility (VaxiJen, AllerTOP, and PepCalc). The final output showed four potentially antigenic, nonallergenic epitopes having good water solubility, comprising “TQKNDGDG” (antigenicity score: 1.5354), “KEDGHTQK” (antigenicity score: 1.2394), “AQEKNEDGHNVGD” (antigenicity score: 1.1338), and “GDGPKEGENLQ” (antigenicity score: 1.2153). Moreover, three conformational B-cell epitopes with populated residues were predicted for this protein using the ElliPro tool, which is involved in antigen-antibody interactions.

Given the intracellular nature of *Leishmania* parasites, helper type-1 CD_4_^+^ (Th1) and cytotoxic CD_8_^+^ T-cells (CTLs) are key regulators in controlling leishmaniasis. Moreover, the capability of IFN-*γ* induction is a pivotal function for Th1-type epitopes, resulting in the activation of macrophages and downstream parasite clearance mechanisms [61]. It has been shown that rHASPB can induce protective immunity against *L. donovani* infection via direct and/or indirect interleukin-12 (IL-12) production and subsequent CD_8_^+^-dependent IFN-*γ* induction [62]. Moreover, several viral vector-based (adenovirus and lentivirus) fusion protein vaccines have, also, demonstrated significant humoral and cellular (IFN-*γ* and IL-4) immune responses against *L. major* [63], *L. donovani* [64], and *L. infantum* [19]. On this basis, further attention should be paid to the epitope analysis of LdHASPB1. In the current study, specific human HTL and CTL epitopes along with the dog CTL epitopes were predicted and screened in terms of antigenicity, allergenicity, and IFN-*γ* induction. Of note, predicted HTL epitopes were mostly located at positions 23-39. Potent human IFN-*γ* inducing HTL epitopes predicted by the IEDB server was in association with the HLA-DQA1^∗^05 : 01/DQB1^∗^03 : 01, as one of the prevalent HLA alleles, including “EANHGGATGVPPKHT” (antigenicity score: 0.9030) and “TEANHGGATGVPPKHT” (antigenicity score: 1.0112). Among human CTL epitopes, five were selected as potentially antigenic and nonallergenic ones, based on the IEDB HLA reference set covering over 97% of the population, enclosing “EANHGGATGV” (HLA-A_∗_68 : 02), “EPQKRADNI” (HLA-B^∗^51 : 01), “SAKEPQKRA” (HLA-A^∗^30 : 01), “APKEDGHTQ” (HLA-B^∗^07 : 02), and “EPQKRADNI” (HLA-B^∗^08 : 01). Since dogs are important reservoirs of *L. donovani* in the Old World countries, CTL epitope analysis for LdHASPB1 was, also, done regarding DLA, using the IEDB server. Our results suggested five high-ranked antigenic and nonallergenic epitopes regarding DLA class-I molecules, such as “KDSAKEPQKR” (DLA-8803401), “EANHGGATGV,” and “KTTEANHGGA” (DLA-8850101), as well as “KDSAKEPQKR” and “TQKNDGDGPK” (DLA-8850801). Altogether, the clinical implications of these specific B- and T-cell epitopes can be assigned to design and engineer different and novel multiepitope vaccine constructs using the predicted epitopes and those of other highly immunogenic *Leishmania* proteins, along with a Th1-biasing adjuvant such as the RS-09 synthetic protein (toll-like receptor 4 agonist) for enhanced immunogenicity. The major challenge in designing such vaccine candidates may be their *in vivo* safety and reliability, which need to be further evaluated using wet experimental methods against human or canine challenges with VL.

## 5. Conclusion

Due to the importance of VL in tropical and subtropical regions and its zoonotic aspects, preventive measures such as vaccination seem to be more effective than therapeutic approaches. Next-generation vaccine design using strictly screened, highly antigenic epitopic fragments of known *L. donovani* antigens in the context of unprecedented immunization platforms provides novel insights into the vaccination against kala-azar. In the present study, the most functional and important biophysical properties and novel B- and T-cell-binding epitopes were predicted in the LdHASPB1 protein of *L. donovani* using a set of immunoinformatic servers. Notably, several CTL epitopes were predicted for human HLA reference alleles and three DLA class-I alleles, which could be further allocated in vaccination studies against VL, as alone or combined with other epitopes/antigens, in the context of a multiepitope vaccine. As a final word, the information provided here, particularly the immunogenic CTL, HTL, and B-cell epitopes, can be of interest to vaccinology researchers and may give insight for designing novel vaccines against VL.

## Figures and Tables

**Figure 1:** Prediction of the secondary structure LdHASPB1 protein using the NetSurfP-3.0 server, showing exposed regions (first line), predominant coils (second line), and disordered regions (third line) below sequences. Thickness of the gray line shows the higher probability of disordered regions.

**Figure 2:** The homology modelling of tertiary structure of LdHASPB1 using the I-TASSER server.

**Figure 3:** Improvement validations in the refined model (*Z*-score: -1), in comparison with the crude model (*Z*-score: -0.77), using the ProSA-web tool.

**Figure 4:** Ramachandran plot analysis of the refined model, in comparison with the crude model. In the crude model, 165 (56.3%), 91 (31.1%), 22 (7.5%), and 15 (5.1%) of the residues were assigned to the most favored, additional allowed, generously allowed, and disallowed regions, respectively, whereas in the refined model, 216 (73.7%), 55 (18.8%), 8 (2.7%), and 14 (4.8%) of residues belonged to the most favored, additional allowed, generously allowed, and disallowed regions, respectively.

**Figure 5:** Conformational B-cell epitopes for the LdHASPB1 protein, predicted using the ElliPro tool of the IEDB server; they consist of (1) 14 residues (score: 0.802), (2) 107 residues (score: 0.695), and (3) 105 residues (score: 0.679).

**Table 1:** Prediction of different characteristics of *L. donovani* HASPB1, using different immunoinformatics web servers.

*In silico* predicted parameters	Used servers and web addresses	*L. donovani* HASPB1
Antigenicity	VaxiJen v2.0, http://www.ddg-pharmfac.net/vaxijen/	1.4409
Allergenicity	AlgPred v2.0, https://webs.iiitd.edu.in/raghava/algpred2/	Yes
Protein solubility	Protein-sol, https://protein-sol.manchester.ac.uk/	0.749 (highly soluble)
Number of residues	ExPASy ProtParam, https://web.expasy.org/protparam/	401
Molecular weight		42196.62
pI		4.64
Positively charged residues (Arg+Lys)		53
Negatively charged residues (Asp + Glu)		106
Half-life in mammalian reticulocytes		30 hours
Instability index		21.34 (stable)
Aliphatic index		5.89
GRAVY score		-2.322 (highly hydrophilic)
Signal peptide	SignalP-6.0, https://services.healthtech.dtu.dk/service.php?SignalP-6.0	No signal peptide (sec/SPI)
Transmembrane domain	DeepTMHMM, https://dtu.biolib.com/DeepTMHMM	No (most likely globular)
Subcellular localization	DeepLoc2.0, https://services.healthtech.dtu.dk/service.php?DeepLoc-2.0	Cell membrane (0.63)
N-Glycosylation	NetNGlyc-1.0, https://services.healthtech.dtu.dk/service.php?NetNGlyc-1.0	Single site at position 44
O-Glycosylation	NetOGlyc-4.0, https://services.healthtech.dtu.dk/service.php?NetOGlyc-4.0	16 sites at positions 3, 4, 6, 9, 23, 24, 32, 39, 41, 46, 96, 110, 124, 180, 320, and 334
Palmitoylation	CSS-palm, http://csspalm.biocuckoo.org/	Single site at position 5
Serine (S), threonine (T), and tyrosine (Y) phosphorylation	NetPhos-3.1, https://services.healthtech.dtu.dk/service.php?NetPhos-3.1	28 sites at positions: 4, 9, and 36 (S); 6, 23, 32, 54, 68, 82, 96, 110, 124, 138, 152, 166, 180, 194, 208, 222, 236, 250, 264, 278, 292, 306, 320, 334, and 348 (T)
Lysine acetylation	GPS-PAIL, http://pail.biocuckoo.org/	11 sites at positions 7, 11, 15, 22, 63, 77, 91, 105, 119, 133, and 147
Secondary structure	NetSurfP-3.0, https://services.healthtech.dtu.dk/service.php?NetSurfP-3.0	Exposed residues in most sites, coils are frequent with a high probability of disordered regions
Tertiary structure (3D model)	I-TASSER, https://zhanggroup.org/I-TASSER/	*C*-score: -0.79, estimated TM-score: 0.61 ± 0.14, estimated root-mean-square deviation (RMSD): 8.6 ± 4.5 Å

**Table 2:** The final screening of shared linear B-cell epitopes from the LdHASPB1 protein.

Shared B-cell epitopes	VaxiJen antigenicity score	AllerTOP allergenicity prediction	PepCalc water solubility prediction
KEDGHTQKNDG	1.3843	Yes	Weak
TQKNDGDG^∗^	1.5354	No	Good
KEDGHTQK^∗^	1.2394	No	Good
PQKRADN	0.5911	No	Weak
AQEKNEDGHNVGD^∗^	1.1338	No	Good
IHKTTEANH	0.2796	Yes	Good
PKEDGHTQK	1.2709	No	Weak
GDGPKEGENLQ^∗^	1.2153	No	Good

^∗^Potent shared antigenic and allergenic linear B-cell epitopes with good water solubility.

**Table 3:** Human helper T-lymphocyte (HTL) epitope prediction for LdHASPB1 using the IEDB HLA reference set, with subsequent screening regarding antigenicity, allergenicity, and IFN-*γ* induction.

Allele	HTL epitope	Method	Percentile rank	Antigenicity	Allergenicity	IFN-*γ* inducer
HLA-DQA1^∗^05 : 01/DQB1^∗^03 : 01	TEANHGGATGVPPK	Consensus (comb.lib./smm/nn)	2.00	1.1249	No	Negative
HLA-DQA1^∗^05 : 01/DQB1^∗^03 : 01	TTEANHGGATGVPP	Consensus (comb.lib./smm/nn)	2.1	1.1017	No	Negative
HLA-DQA1^∗^05 : 01/DQB1^∗^03 : 01	TEANHGGATGVPP	Consensus (comb.lib./smm/nn)	1.6	1.0977	No	Negative
HLA-DQA1^∗^05 : 01/DQB1^∗^03 : 01	KTTEANHGGATGVPP	Consensus (comb.lib./smm/nn)	2.6	0.9802	No	Negative
HLA-DQA1^∗^05 : 01/DQB1^∗^03 : 01	TEANHGGATGVPPKH	Consensus (comb.lib./smm/nn)	2.6	1.1819	Yes	Negative
HLA-DQA1^∗^05 : 01/DQB1^∗^03 : 01	TTEANHGGATGVPPK	Consensus (comb.lib./smm/nn)	2.6	1.1256	Yes	Negative
HLA-DQA1^∗^05 : 01/DQB1^∗^03 : 01	ANHGGATGVPPKHT	Consensus (comb.lib./smm/nn)	2.5	0.7527	Yes	Negative
HLA-DQA1^∗^05 : 01/DQB1^∗^03 : 01	EANHGGATGVPPKHT	Consensus (comb.lib./smm/nn)	2.8	0.9030	No	Positive
HLA-DQA1^∗^05 : 01/DQB1^∗^03 : 01	EANHGGATGVPPKH	Consensus (comb.lib./smm/nn)	2.9	1.0807	No	Negative
HLA-DQA1^∗^05 : 01/DQB1^∗^03 : 01	TEANHGGATGVPPKHT	Consensus (comb.lib./smm/nn)	2.7	1.0112	No	Positive

**Table 4:** Human cytotoxic T-lymphocyte (CTL) epitope prediction for LdHASPB1 using the IEDB HLA reference set, with subsequent screening in terms of antigenicity and allergenicity.

HLA allele	Epitope length	Sequence	Percentile rank: <1	Antigenicity	AllerTOP allergenicity
HLA-B^∗^07 : 02	10	VPPKHTGSAM	0.04	0.2065	Yes
HLA-A^∗^68 : 01	9	DSAKEPQKR	0.2	1.3388	Yes
HLA-B^∗^07 : 02	9	PPKHTGSAM	0.18	0.3758	No
HLA-A^∗^11 : 01	9	SAMNDSAPK	0.25	0.7898	Yes
HLA-A^∗^33 : 01	9	DSAKEPQKR	0.26	1.3388	Yes
HLA-B^∗^07 : 02	9	VPPKHTGSA	0.35	0.1872	Yes
HLA-A^∗^68 : 01	9	SAMNDSAPK	0.97	0.7898	Yes
HLA-A^∗^68 : 02	10	EANHGGATGV^∗^	0.34	1.1771	No
HLA-A^∗^11 : 01	10	GSAMNDSAPK	0.52	1.3978	Yes
HLA-A^∗^11 : 01	9	GGATGVPPK	0.53	0.5969	Yes
HLA-A^∗^30 : 01	9	SAMNDSAPK	0.52	0.7898	Yes
HLA-B^∗^51 : 01	9	EPQKRADNI^∗^	0.56	0.7975	No
HLA-A^∗^30 : 01	9	GGATGVPPK	0.56	0.5969	Yes
HLA-B^∗^44 : 03	10	QEKNEDGHNV	0.49	1.1248	Yes
HLA-B^∗^44 : 02	10	QEKNEDGHNV	0.44	1.1248	Yes
HLA-B^∗^35 : 01	10	VPPKHTGSAM	0.6	0.2065	Yes
HLA-A^∗^30 : 01	9	SAKEPQKRA^∗^	0.75	1.5432	No
HLA-B^∗^07 : 02	9	APKEDGHTQ^∗^	0.7	1.5982	No
HLA-B^∗^08 : 01	9	EPQKRADNI^∗^	0.67	0.7975	No

^∗^The final qualified epitopes regarding percentile rank, antigenicity, and allergenicity.

**Table 5:** Dog leukocyte antigen (DLA) class-I epitope prediction for LdHASPB1 using the IEDB server, with subsequent screening in terms of antigenicity and allergenicity.

DLA allele	Position	Sequence	Percentile rank	Antigenicity	AllerTOP allergenicity
DLA-8803401	33-42	GVPPKHTGSA	11	0.2291	Yes
	3-12	QQNDGDAQEK	11	1.2084	Yes
	7-16	KDSAKEPQKR^∗^	12	1.5395	No
	34-43	VPPKHTGSAM	13	0.2065	Yes
	29-38	GGATGVPPKH	14	0.7968	Yes

DLA-8850101	33-42	GVPPKHTGSA	6.9	0.2291	Yes
	34-43	VPPKHTGSAM	11	0.2065	Yes
	3-12	QQNDGDAQEK	14	1.2084	Yes
	25-34	EANHGGATGV^∗^	17	1.1771	No
	22-31	KTTEANHGGA^∗^	21	1.0364	No

DLA-8850801	3-12	QQNDGDAQEK	1.3	1.2084	Yes
	7-16	KDSAKEPQKR^∗^	2.8	1.5395	No
	48-57	TQKNDGDGPK^∗^	5.5	0.7858	No
	34-43	TQKNDGDGPK	5.5	0.7858	No
	20-29	TQKNDGDGPK	5.5	0.7858	No

^∗^The final qualified epitopes regarding percentile rank, antigenicity, and allergenicity.

## Data Availability

The data used to support the findings of this study are available from the corresponding author upon request.
